# Quantifying Region-Specific Elastic Properties of Distal Femoral Articular Cartilage: A Shear-Wave Elastography Study

**DOI:** 10.1155/2022/9406863

**Published:** 2022-02-07

**Authors:** Weixin Deng, Ming Lin, Suiqing Yu, Hongying Liang, Zhijie Zhang, Chunlong Liu

**Affiliations:** ^1^Clinical College of Acupuncture, Moxibustion and Rehabilitation, Guangzhou University of Chinese Medicine, Guangzhou, China; ^2^Luoyang Orthopedic Hospital of Henan Province, Orthopedic Hospital of Henan Province, Luoyang, China

## Abstract

Knee osteoarthritis is a disease with the degeneration of articular cartilage as its main feature. Cartilage thickness cannot become a single index to evaluate cartilage degeneration, so it is essential to also evaluate the stiffness. The purposes were as follows: (1) to examine test-retest reliabilities of the elastic modulus measurement in distal femoral articular cartilage (FAC) and compare the changes in specific-regional of distal FAC, (2) to explore the difference in distal FAC stiffness and thickness between the dominant and nondominant sides, and (3) to examine the correlation between the elastic properties of cartilage and the thickness of cartilage. Twenty healthy participants were recruited. The stiffness of distal FAC at the lateral femoral condyle (LFC), medial femoral condyle (MFC), and intercondylar notch (IN) was quantified using shear-wave elastography (SWE). Intra- and interrater reliabilities were excellent for measuring the stiffness of distal FAC (ICC: 0.83-0.98). About a 50% increase in the stiffness of LFC (40.78 kPa) was found when compared with IN (21.82 kPa) and MFC (18.34 kPa). No significant difference was found between the dominant and nondominant sides in distal FAC stiffness and thickness. There was no correlation between the stiffness and thickness of the distal FAC. In conclusion, SWE can quantify the stiffness of the distal FAC.

## 1. Introduction

Osteoarthritis (OA) is the most common form of arthritis and one of the leading causes of chronic disability in the elderly population worldwide [1–3]. The knee joint is composed of osseous structures, cartilage, ligaments, and a synovial membrane [2]. With high use and stress on the knee, it is one of the most frequently affected sites by OA. Knee OA (KOA) is a disease with the degeneration of articular cartilage as one of its main features [3, 4]. The main risk factors associated with KOA are obesity, previous knee trauma, hand OA, female gender, and age [5]. As part of the onset of OA, excessive physiological load causes the extracellular matrix to become compromised or the synthesis of components to become reduced, resulting in increased stress on chondrocytes, which may cause cell death [6]. In another way, the increasing activity or production of proinflammatory cytokines causes the content of proteoglycans to decrease, resulting in cartilage deformation in response to loading. A reduced amount of proteoglycans is related to the decreasing stiffness of the cartilage. Losing proteoglycans may affect the cartilage's ability to experience and transfer stress [7]. Due to the viscoelasticity of cartilage and repeated loading, cartilage deformation cannot be restored completely [8]. Although there are many methods for treating KOA, as of now, pain is the biggest perplexing problem for patients. In the early phase of KOA, the cartilage is thicker due to swelling or hypertrophy [9]. However, neuropathic pain has not been associated with cartilage thickness [10]. Therefore, cartilage thickness cannot become a single index for evaluating cartilage degeneration. The quantification of the elastic properties of distal FAC is essential for gaining insight into the degeneration of articular cartilage [11]. Early detection of KOA is needed to delay the progression and minimize cartilage degeneration. Thus, it is important to evaluate the stiffness of the cartilage. The diagnosis of KOA occurs through clinical evaluation, which is supplemented by conventional radiology. X-rays illustrate the bony abnormalities of osteoarthritis but fail to directly visualize articular cartilage. There are several ways to assess the elastic properties of cartilage. Magnetic resonance elastography has been proven to be a capable tool for assessing the stiffness of baboon intervertebral discs ex vivo [12]. Optical Fiber Polarimetric Elastography (OFPE) can also be used for the biomechanical analysis of porcine cartilage elasticity [13]. One study found different cartilage elasticities between smokers and nonsmokers by using real-time sonoelastography to measure strain ratios [14]. Similarly, another study showed that real-time sonoelastography may be a useful tool for detecting early changes in cartilage stiffness after anterior cruciate ligament reconstruction [15]. Arthroscopy can directly inspect the surface of articular cartilage but is invasive [16].

More recently used, SWE is an ultrasound elastography technology for easily and noninvasively quantifying the elastic properties of tissue [17, 18]. It generates shear waves through an acoustic radiation force that propagates through the surrounding tissue and traces the wave back to provide biomechanical information about the tissue of the measured object [19, 20]. It is widely used for muscles, ligaments, and tendons [21]. One recent study has demonstrated that SWE is a feasible method for quantifying the elastic properties of lower lateral nasal cartilage, costal cartilage, and conchal cartilage [22]. Few studies have been conducted to investigate the specific-regional elastic properties of distal FAC.

Therefore, the aims of the study were as follows: (1) to assess the intra- and interrater reliabilities of the elastic modulus measurement in distal FAC and compare changes in specific-regional of distal FAC, (2) to investigate differences in distal FAC stiffness and thickness between the dominant and nondominant sides, and (3) to investigate the relationship between the elastic properties of cartilage and the thickness of cartilage.

## 2. Materials and Methods

### 2.1. Participants' Recruitment

Participants were included if they were healthy (no comorbidities, no joint pain) and could follow the instructions of the rater. The exclusion criteria were as follows: knee ligament injury, chronic ankle instability, knee pain or discomfort for 6 months before the experiment, a history of severe trauma, or knee surgery [14, 23, 24]. Participants were prohibited from exercising for 48 hours before the experiment. Twenty participants (ten males and ten females) were recruited for the study. Demographic information, including age and body mass index (BMI) for all participants, is shown in Table 1.

### 2.2. Experimental Procedures

This experiment was an observational study. The knee was fixed on a quadriceps femoris exercise board with 120° of flexion assessed by a joint goniometer (Figure 1(a)). The stiffness and thickness of the distal FAC were measured by an ultrasound (US) device. Two raters (DWX and LM) took part in the interrater investigation. In the first test, two raters took turns examining the distal FAC of each participant. Participants were asked to attend the second test at the same time as the first test, 5 days later, and the test was conducted by rater DWX for the intrarater investigation. Participants were asked to maintain their normal activity but to avoid additional activity [25]. The dominant leg of participants was determined by kicking a ball [26].

### 2.3. Equipment

The shear modulus of the knee joint was quantified using the ultrasound shear wave elastography system with a 40 mm linear array transducer (SL10-2, Aixplorer SuperSonic Imagine, France). The settings were as follows: the frequency was 2-10 MHz. The opacity was set to 85% [26]. The measurable range of elastic modulus was 0-100 kPa. The color scale used in the shear modulus (in kPa) showed the lowest values in blue and the highest values in red.

Ultrasound joint examination was performed using light pressure and a large quantity of visible scanning gel between the transducer and the skin [27]. Once the distal FAC was identified, the probe was aligned and parallel to the distal FAC, and the SWE mode was activated to measure the distal FAC shear elastic modulus. The same model and machine were used for all participants. Before testing, participants could have a 5-minute rest in a supine position. The temperature in the room was kept at 25°C [26]. The transducer was placed transversely to the leg above the superior margin of the patella. When the midpoint of the intercondylar notch was imaged at the center of the machine screen, one rater marked two lines on the knee skin, each one at the midpoint of the lateral edges of the transducer. The transducer was placed between the two lines marked on the skin. The mark on the knee skin was to help find the approximate location of the distal FAC.

### 2.4. Quantifying the Elastic Properties of Distal FAC

To assess the stiffness of the distal FAC, the knee was flexed to 120°. It was reported that 120° for measuring distal FAC could be successfully performed by every patient [28, 29]. The knee was supported on a quadriceps femoris exercise board to keep the leg in neutral alignment in the coronal and transverse planes. The probe was stationed on the skin perpendicularly for 8–12 seconds [30]. The points where the line drawn on the transparent sheet intersected the bone-cartilage interface at the LFC, MFC, and IN were taken as reference US measurement points [31]. Three images were captured of each site [32]. The images were saved when the color in the region of interest (ROI) was uniform and were stored for offline analysis. Offline analysis was conducted using elasticity maps, which are expressed in kPa (Figures 1(c)–1(e)). The difference between the SWE mode and the B-mode is that an acquisition box appears in the SWE mode. The elastic map generated in SWE mode is a real-time color change image in the acquisition box superimposed on the B-mode image. The acquisition box moved to IN, LFC, or MFC and then fixed it. The region of interest (ROI) is a moveable circle inside the acquisition box to describe the elastic modulus in that circle area. The diameter of the ROI was set to the minimum value of 1 mm. The Q-Box™, which is displayed on the right side of the screen, represents the average, minimum, maximum, and SD values in the ROI [33].

### 2.5. Quantifying the Thickness of the Distal FAC

Reference US measurement points of distal FAC thickness were perpendicular line distances (cm) that were drawn from the hyperechoic cartilage-bone interface to the synovial space-cartilage interface [34]. The first measurement point was taken at IN. Measurement 2 was the midpoint between IN and MFC. Measurement 3 was the midpoint between IN and LFC [31]. Three images were taken from the right intercondylar notch (RIN), right medial femoral condyle (RMFC), right lateral femoral condyle (RLFC), left intercondylar notch (LIN), left medial femoral condyle (LMFC), and left lateral femoral condyle (LLFC), respectively. The distal FAC status was monitored by an examiner during the capture of the shear-wave imaging map (Figure 1(b))

### 2.6. Statistical Analysis

Statistical analysis was performed using SPSS version 22.0 software (SPSS Inc., Chicago, IL). The Shapiro-Wilk test was used to determine the normality distribution. The Wilcoxon test was used to calculate the shear elastic modulus between dominant and nondominant legs. Pearson's correlation analysis (*r*) was used to examine the correlation of distal FAC between stiffness and thickness. The intra- and interrater reliabilities were evaluated by calculating the intraclass correlation coefficient (ICC) with a 95% confidence interval. The intrarater (measurements taken on two occasions separated by 5 days) and interrater (measurements by two raters) reliability of the measurement of distal FAC stiffness was examined using ICC (3.1) (two-way mixed effects model, consistency) and ICC (2.2) (two-way random effects model, absolute agreement). The standard error of the mean (SEM) was calculated by the formula $\text{SEM}=\text{standard deviation}\times \sqrt{1-\text{ICC}}$, while the minimal detectable change (MDC) was computed by the formula $\text{MDC}=1.96\times \text{SEM}\times \sqrt{2}$ [25]. Bland and Altman plots were used to assess intra- and interrater reliability by determining the degree of agreement. The differences in the shear modulus of distal FAC in IN, MFC, and LFC were analyzed by a one-way repeated measures analysis of variance (ANOVA). If there was statistical significance in the test (*p* < 0.05), an independent *t*-test was used to compare the mean value of each relevant measurement data set, and post hoc Bonferroni testing was performed. Intraclass correlation coefficient values < 0.50 were considered poor, 0.50-0.60 were considered moderate, 0.60-0.80 were considered good, and 0.80-1.0 were considered excellent [33]. For all tests, the statistical significance was set at *p* < 0.05, and all measurement data was expressed as means (standard deviations).

## 3. Results

### 3.1. Intra- and Interrater Reliabilities

Both intra- and interrater reliability for measuring distal FAC stiffness were excellent, with ICC values above 0.80, SEM less than 3 kPa, and MDC less than 7 kPa (Table 2).  Figure 2(a) depicts Bland and Altman plots for interrater reliability, while Figure 2(b) depicts data for intrarater reliability. For intra- and interrater reliability of LIN, the mean difference was 0.51 kPa and 0.34 kPa, respectively, and the 95% limit of agreement (LOA) was from -5.39 kPa to 6.40 kPa and from -3.93 kPa to 4.60 kPa, respectively. For LMFC, the mean difference was -0.41 kPa and 0.27 kPa, and the 95% LOA was from -5.23 kPa to 4.41 kPa and from -1.96 kPa to 2.49 kPa. For LLFC, the mean difference was 0.06 kPa and 0.66 kPa, and the 95% LOA was from -9.41 kPa to 9.53 kPa and from -9.40 kPa to 10.71 kPa. For RIN, the mean difference was -0.13 kPa and 0.73 kPa, and the 95% LOA was from -3.59 kPa to 3.34 kPa and from -2.66 kPa to 4.12 kPa. For RMFC, the mean difference was 0.32 kPa and 0.95 kPa, and the 95% LOA was from -5.90 kPa to 6.53 kPa and from -4.64 kPa to 6.53 kPa. For RLFC, the mean difference was 1.31 kPa and -0.06 kPa, and the 95% LOA was from -8.18 kPa to 10.79 kPa and from -6.01 kPa to 5.90 kPa.

### 3.2. Differences in the Stiffness of MFC, IN, and LFC

The mean stiffness of LIN was 20.65 kPa, that of LMFC was 19.42 kPa, and that of LLFC was 39.73 kPa, while that of RIN was 21.82 kPa, that of RMFC was 18.34 kPa, and that of RLFC was 40.78 kPa. There are comparisons of stiffness between the LIN and the LMFC (*p* = 0.60), the LIN and the LLFC (*p* < 0.01), the LMFC and the LLFC (*p* < 0.01), the RIN and the RMFC (*p* = 0.15), the RIN and the RLFC (*p* < 0.01), and the RMFC and the RLFC (*p* < 0.01) (Figure 3).

### 3.3. Differences in the Stiffness and Thickness of the Distal FAC between the Dominant and Nondominant Sides

There was no significant difference in the elastic modulus and thickness of the distal FAC between the dominant and nondominant sides (Table 3).

### 3.4. The Relationship between the Thickness of the Distal FAC and Its Stiffness

No significant correlation was found between thickness and stiffness on both sides. The *r* values and *p* values of the distal FAC for stiffness and thickness are shown in Table 4.

## 4. Discussion

The most important finding of this study is that SWE is a feasible modality for assessing the shear modulus of the distal FAC in different regions. Intra- and interrater reliabilities for evaluating distal FAC stiffness by using SWE were excellent, with relatively low SEM and MDC values. The relatively low SEM and MDC values in the results may prove the accuracy of the measurement.

In the present study, intra- and interrater reliability of elastic properties ranged from good to excellent for assessing distal FAC, which was consistent with those of previous studies evaluating cartilage. Gungor et al. used sonoelastography to detect the strain ratio measurements of femoral cartilage, and the result was high intraobserver reliability, with an ICC of 0.94 in IN [14]. Another study also observed high intrarater reliability of strain ratio measurements via sonoelastography and for femoral cartilage found 0.97 in IN [15]. To sum up, ultrasound imaging is a repeatable technique for assessing cartilage elasticity. In the present study, the ICC values for interrater reliability were relatively high compared to those for intrarater reliability. Possible explanations might be that the amount of exercise or other factors in the 5-day period influenced the accuracy of the experiment. Another explanation might be the different knee flexion angles. Participants in previous studies were asked to flex their knees to the maximum angle, at least 125 degrees [14, 15, 24, 35]. The findings from this study indicated that SWE is a reliable instrument for quantifying the elastic properties of distal FAC.

The Bland-Altman plots of the present study data further verified the consistency of the findings. As shown in Figure 2, most of the data points were within the 95% confidence limit. Therefore, the consistency of this study's data is satisfactory.

The stiffness of distal FAC in different regions was quantified using SWE in this study. Objective information on the stiffness of different regions of the FAC distal to healthy participants may be useful to clinicians. Furthermore, the cartilage was significantly stiffer in the LFC when compared with that in the MFC and IN. About a 50% increase in the stiffness of the LFC was found when compared with the IN and MFC. It is difficult to directly compare the present findings to those from previous studies of measurement. The range of elastic modulus from the results of this study was similar to a recent study [22]. This study attempted to quantify the elastic properties of auricular conchal cartilage, nasal cartilage, and costal cartilage using SWE. Shear-wave elastography could be quantified by the elastic modulus of lateral nasal cartilage (29.31 kPa), auricular conchal cartilage (28.33 kPa), and costal cartilage (53 kPa). A higher elastic modulus in a costal cartilage was obtained when compared with lateral nasal cartilage and auricular conchal cartilage. In this study, the mean stiffness of the LIN was 20.65 kPa, that of the LMFC was 19.42 kPa, that of the LLFC was 39.73 kPa, that of the RIN was 21.82 kPa, that of the RMFC was 18.34 kPa, and that of the RLFC was 40.78 kPa. Furthermore, previous studies investigating strain found a negative correlation to stiffness [36]. The strain of cartilage correlates with the biomechanics and components of the cartilage itself. Femoral cartilage strain was positively correlated with BMI and body fat percentage. The findings confirmed that one of the KOA risk factors is obesity, in which high BMI and body fat percentage increase strain on femoral cartilage [7]. The more loaded, the softer the cartilage [15]. A high BMI may affect not only joint loading but also the osmotic environment of chondrocytes [8]. A reduction of proteoglycans reflects the degeneration of cartilage. Proteoglycans affect the ability of cartilage to bear weight and transfer loading [7]. Losing proteoglycans can increase the strain on the cartilage and is reflected in the decrease in stiffness. An increased strain ratio in sonoelastography represents softening. The strain ratio of pathologic cartilage was higher than that of normal cartilage [35]. Strain is the relative deformation of the tissue as it responds to pressure. On the basis that the reference strain is relatively constant, the lower the strain of the target tissue, the lower the strain ratio. Since the relative deformation is small when the stiffness is high, the lower the strain of the target tissue, the higher the stiffness and the worse the elasticity. The strain ratio used in strain ultrasound elastography was the ratio of the target tissue strain to the reference strain, which was a measurement of relative stiffness, while the SWE used in this study could obtain a direct stiffness measurement intuitively.

There were no significant differences observed in the elastic modulus or thickness of the distal FAC between the dominant and nondominant sides. The present findings were consistent with previous studies that evaluated the elastic features of the quadriceps tendon and patella tendon in the dominant and non-dominant leg [36]. In this study, all participants used their right leg as the dominant leg. One study showed that lower limb strength was negatively correlated with the strain ratio, which was further related to cartilage stiffness [15]. That means that lower extremity strength may positively correlate with cartilage stiffness. Further studies may be necessary to determine the relationship between lower extremity strength and cartilage stiffness. Another study demonstrated that tissue stiffness was related to cartilage loading [23]. They found that T1 rho and T2 relaxation time decreased after physical activities, in which T1 values were negatively related to proteoglycans and T2 values were positively related to collagen and water content. The cartilage experienced more loading in physical activities, and this was reflected in the reduction of T1 rho and T2 values. The dominant side should be the preferred side, so it should be used more than the nondominant side. Therefore, there should be a difference in lower limb strength and load-bearing capacity, but the present research found that this is not the case. The difference between the dominant side and the nondominant side was not significant. Further analysis revealed that the gender difference between the dominant side and the nondominant side was also not significant.

Then explore the potential gender impact. Age and BMI showed no significant differences between the genders. Interestingly, no significant difference in stiffness was observed between males and females in all test regions (all *p* values > 0.05), but a significant difference in thickness was observed between males and females in all test regions (all *p* values < 0.05) except RIN. For stiffness, no significant difference was found between the dominant side and the non-dominant side, regardless of whether they were male or female. For thickness, a significant difference was found at IN in females between the dominant side and the nondominant side. However, different sports and doses affect stress on cartilage. Normal walking for 20 minutes causes significant strains on the articular cartilage [37]. After 30 minutes of walking, running, or sitting, cartilage deformation has been observed in both walking and running groups [24]. Cartilage deformation indicates that changes may happen in the stiffness of cartilage. However, Harkey et al. [24] only examined the thickness of cartilage rather than stiffness. Compared to the present study, cartilage stiffness was only examined at a static status rather than after exercising. Each subject's daily exercise methods, time, intensity, and frequency were different. For example, among male subjects, there were differences in basketball, football, running, etc., while among female subjects, there were differences in rope skipping, yoga, etc. Long-term accumulation of exercise, including exercise type, intensity, etc., will affect the distal FAC. This can explain why the range of elastic modulus of the distal FAC of the subjects fluctuated within a certain range. Each subject chose multiple compound exercises instead of a single exercise. Thus, it is impossible to conclude which types of sports will affect the more distal FAC.

In addition, it was found that there was a negative correlation between BMI and MFC (dominant side) (*r* = −0.47, *p* = 0.04), which was consistent with previous studies and proved that BMI was one risk factor for KOA. On this basis, it seems to further prove that BMI was related to MFC on the dominant side. Unfortunately, there were no participants in this study whose left side was the dominant side.

The validity of US for assessing the thickness of distal FAC has been proven [31]. In the present study, no significant correlation was found between the thickness and stiffness of the distal FAC. Similarly, the comparison after separating the genders also had no significant correlation (all *p* values > 0.05). In the view of biomechanics, when the cartilage is pressed, the fluid in the cartilage flies out, which results in a thinner cartilage [38]. With less fluid within the cartilage, the stiffness of the cartilage may increase. Inflammatory factors such as TNF- and IL-1 can be reduced through diet and exercise [39]. Increasing the vitality of those factors results in the reduction of proteoglycans, which can decrease the stiffness of cartilage. A reduction of proteoglycans may contribute to the decrease in the thickness of cartilage. At different stages of KOA, the thickness of the cartilage changes. The early degeneration of cartilage becomes thicker due to swelling or hypertrophy [9]. The participants in this study were healthy young subjects, not KOA patients, so it may not be possible to conclude that there is a correlation between cartilage stiffness and thickness. Further studies can continue to study whether there is a correlation between cartilage stiffness and thickness in the KOA patient population. In B-mode ultrasound, the thickness was observed but could not be distinguished as normal or abnormal. In SWE mode, normal or abnormal tissue may be identified by different stiffness levels [14]. Thus, SWE may be used in clinical practice for discovering cartilage disorders, and it is a feasible tool for clinicians to consider not only thickness but also stiffness.

There were several limitations to this study. First, the sample size was small. Second, resting for 45 minutes was advised for the cartilage to relax and return to its original size [38]. Fluid shifts are related to cartilage loading [23]. Participants had only 5 minutes of rest before the evaluation. Thus, the activities before they arrived at the destination and insufficient resting time may have affected the stiffness of their articular cartilage. Finally, all healthy subjects were recruited for the study. Further studies will be conducted to examine the changes in distal FAC between subjects with knee osteoarthritis and elderly and healthy subjects.

## 5. Conclusion

Shear-wave elastography is a noninvasive modality for assessing distal FAC stiffness and detecting side-to-side differences. This information allows clinicians to clearly understand the relationship between distal FAC elastic properties and clinical manifestations. Although a relationship between thickness and stiffness in healthy participants was not found, further studies may help investigate the stiffness of distal FAC using SWE among knee osteoarthritis patients and the elderly healthy population.

## Figures and Tables

**Figure 1:** (a) The participant was supine, with one knee fixed on a quadriceps femoris exercise board at 120° of flexion. (b) B-mode maps for measuring the thickness of the distal FAC. (c–e): SWE maps for measuring the stiffness of the distal FAC. Upper images: color-coded box presentations of distal FAC elasticity were shown (the image color represents stiffness: blue represents soft while red represents stiff). Lower images: B-mode images of the distal FAC. The Q-Box™ is shown on the right. IN: intercondylar notch; MFC: medial femoral condyle; LFC: lateral femoral condyle.

**Figure 2:** Bland and Altman plots of intra- and interrater reliability of distal FAC stiffness. The difference of IN, MFC, and LFC in distal FAC stiffness between rater DWX and rater LM was plotted against the mean distal FAC stiffness (average of the 2 raters) for each participant (a). The difference of IN, MFC, and LFC in distal FAC stiffness between day 1 and day 5 was plotted against mean distal FAC stiffness (average of the days for rater DWX) for each participant (b). In each panel, the continuous line represents the mean difference, and the dotted lines represent 2 SD above and below the mean difference.

**Figure 3:** Comparisons of stiffness between specific regions of distal FAC. ∗ means a significant difference.

**Table 1:** Participant's demographic information.

	Male (*n* = 10)	Female (*n* = 10)	Total (*n* = 20)
Age (years)	20.10 ± 1.29	19.60 ± 1.27	19.85 ± 1.27
BMI (kg/m^2^)	20.93 ± 2.28	20.16 ± 2.06	20.55 ± 2.15

The data was displayed as the mean ± SD. SD: standard deviation.

**Table 2:** Inter- and intrarater reliability of IN, MFC, and LFC stiffness.

		Rater DWX in test 1	Rater DWX in test 2	Rater LM	ICC^a^ (95% CI)	ICC^b^ (95% CI)
IN (L)	Mean ± SD (kPa)	20.65 ± 6.92	20.15 ± 7.17	20.08 ± 7.42	0.91 (0.78-0.96)	0.96 (0.89-0.98)
	MDC (kPa)	4.29	4.44	4.60		
	SEM (kPa)	1.55	1.60	1.66		
IN (R)	Mean ± SD (kPa)	21.82 ± 7.54	21.94 ± 8.32	21.17 ± 7.72	0.98 (0.94-0.99)	0.97 (0.93-0.99)
	MDC (kPa)	4.67	5.15	4.78		
	SEM (kPa)	1.69	1.86	1.73		
MFC (L)	Mean ± SD (kPa)	19.42 ± 5.67	19.83 ± 5.51	19.38 ± 5.53	0.90 (0.77-0.96)	0.98 (0.95-0.99)
	MDC (kPa)	3.52	3.41	3.44		
	SEM (kPa)	1.27	1.23	1.24		
MFC (R)	Mean ± SD (kPa)	18.34 ± 7.34	18.02 ± 7.01	17.25 ± 7.39	0.90 (0.77-0.96)	0.92 (0.81-0.97)
	MDC (kPa)	4.55	4.34	4.58		
	SEM (kPa)	1.64	1.57	1.65		
LFC (L)	Mean ± SD (kPa)	39.73 ± 8.83	39.67 ± 9.98	39.05 ± 9.91	0.87 (0.70-0.96)	0.86 (0.68-0.94)
	MDC (kPa)	5.47	6.19	6.14		
	SEM (kPa)	1.97	2.23	2.22		
LFC (R)	Mean ± SD (kPa)	40.78 ± 7.62	39.48 ± 9.12	40.19 ± 9.73	0.83 (0.63-0.93)	0.94 (0.87-0.98)
	MDC (kPa)	4.72	5.65	6.03		
	SEM (kPa)	1.70	2.04	2.18		

L: left sides; R: right sides; IN: intercondylar notch; MFC: medial femoral condyle; LFC: lateral femoral condyle; SD (kPa): standard deviation of kPa; ICC: intraclass correlation coefficient; 95% CI: 95% confidence interval; MDC (kPa): minimal detectable change of kPa; SEM (kPa): standard error of measurement of kPa; kPa: kilo Pascal. ^a^Intrarater reliability. ^b^Interrater reliability.

**Table 3:** Differences in the stiffness and thickness of FAC between dominant and nondominant sides.

	Dominant	Nondominant	*p* value
Thickness (cm)			
IN	0.24 ± 0.06	0.23 ± 0.06	0.29
MFC	0.20 ± 0.04	0.20 ± 0.04	0.77
LFC	0.19 ± 0.04	0.19 ± 0.04	0.51
Stiffness (kPa)			
IN	26.02 ± 16.36	21.71 ± 10.16	0.53
MFC	18.89 ± 8.84	20.25 ± 5.71	0.58
LFC	41.50 ± 16.01	41.75 ± 14.29	0.68

The data was displayed as the mean ± SD. SD: standard deviation.

**Table 4:** Relationship between thickness and stiffness.

	Nondominant	Dominant
MFC	-0.17/0.48	0.32/0.16
IN	-0.05/0.84	-0.30/0.21
LFC	-0.07/0.77	0.29/0.22

The data was presented as *r* and *p* values.

## Data Availability

The data used to support the findings of this study are included within the article.
